The article "Modulation in the Stiffness of Specific Muscles of the Quadriceps in Patients With Knee Osteoarthritis and Their Relationship With Functional Ability" was published in 2022. Journal: Front Bioeng Biotechnol.

# Modulation in the Stiffness of Specific Muscles of the Quadriceps in Patients With Knee Osteoarthritis and Their Relationship With Functional Ability

**DOI:** 10.3389/fbioe.2021.781672

**Published:** 2022-02-10

**Authors:** Tian-Tian Chang, Yuan-Chun Zhu, Zhe Li, Feng Li, Ya-Peng Li, Jia-Yi Guo, Xue-Qiang Wang, Zhi-Jie Zhang

**Affiliations:** ^1^ Rehabilitation Therapy Center, Luoyang Orthopedic Hospital of Henan Province, Orthopedic Hospital of Henan Province, Luoyang, China; ^2^ Department of Sport Rehabilitation, Shanghai University of Sport, Shanghai, China; ^3^ The First Clinical Medical School, Shaanxi University of Chinese Medicine, Xi’an, China; ^4^ Department of Rehabilitation Medicine, Shanghai Shangti Orthopaedic Hospital, Shanghai, China

**Keywords:** stiffness, quadriceps, osteoarthritis, knee, vastus lateralis, WOMAC

## Abstract

Deficits in the flexibility of the quadriceps are one of the risk factors for developing knee joint disorders. No studies have investigated the changes in the stiffness of the quadriceps muscle among patients with knee osteoarthritis (OA). Therefore, the purpose of this study was to investigate changes in the stiffness of specific-muscle of the quadriceps in patients with knee OA and their relationship with functional ability. Twenty-five patients with knee OA and 25 healthy, asymptomatic subjects were recruited in this study. The stiffness of the vastus lateralis (VL), vastus medialis (VM) and rectus femoris (RF) in all participants was evaluated using MyotonPRO at 60° and 90° flexion of the knee joint. The results of this study showed a greater VL stiffness in patients with knee OA than in healthy subjects at both 60° and 90° of knee flexion (*p* < 0.05). Significant differences in VL, VM and RF stiffness were obtained at different knee joint angles in individuals with and without knee OA (*p* < 0.05). In addition, there was a positive correlation between VL stiffness and the Western Ontario and McMaster Universities Osteoarthritis Index (WOMAC) scores in patients with Knee OA (60° of knee flexion: *r* = 0.508, *p* = 0.010; 90° of knee flexion: *r* = 0.456, *p* = 0.022). These results indicate that there is an increase in VL stiffness in patients with knee OA compared with healthy, asymptomatic subjects, and the quadriceps stiffness was increased with knee flexion in both healthy subjects and patients with knee OA. VL stiffness is associated with WOMAC scores in patients with knee OA.

## Introduction

Osteoarthritis (OA) is the most common joint disorder around the world and it can affect many joints but most frequently occurs in the knee (Du et al., 2019). Knee osteoarthritis, characterized by knee joint degeneration, usually occurs during middle to older age (Michael et al., 2010). It is estimated that approximately 37% of individuals (aged > 45 years) are affected by knee OA (Dillon et al., 2006). Furthermore, the prevalence of knee OA has increased because of the increasingly older and obese population worldwide (Hunter and Bierma-Zeinstra, 2019). As a result, knee OA results in a significant social and economic burden (Liu Q et al., 2018). The costs of medical care, indirect costs due to work loss and premature retirement caused by knee OA are escalating (Cross et al., 2014; Safiri et al., 2020). There are many risk factors for knee OA, including a high body mass index (BMI), quadriceps weakness, frequent kneeling and squatting, and participation in sports (Simic et al., 2021; Szilagyi et al., 2021).

The quadriceps muscle plays an important role in shock absorption and knee joint stability during walking and running (Davis et al., 2019; Ebihara et al., 2020). The reduced flexibility of the quadriceps may be one of the risk factors for the development of anterior knee pain, including patellofemoral pain syndrome and patellar tendinopathy, and tight quadriceps muscles may contribute to increasing knee joint stress during functional activities (Witvrouw et al., 2000; Witvrouw et al., 2001; Piva et al., 2005). Previous studies have used the knee range of motion to reflect the flexibility of the quadriceps in patients with knee OA (Cho et al., 2015; Lu et al., 2018; Perlman et al., 2019). However, this method is used to quantify the flexibility of groups of muscles, not individual muscles. The joint range of motion is influenced not only by skeletal muscle but also by noncontractile structures such as skin, tendons and the joint capsule (Geertsen et al., 2015; Andrade et al., 2016; Nordez et al., 2017). Thus, the method used to quantify the joint range of motion could not provide insight into changes in the stiffness of individual muscles. Furthermore, several studies have demonstrated that the stiffness of each individual muscle may be influenced by various factors, such as contraction (Avrillon et al., 2018), stretching (Hirata et al., 2016) and pathology (Zhang et al., 2014; Zhou et al., 2020). In recent years, some studies compared the difference in the stiffness of soft tissues between healthy subjects and patients with musculoskeletal disorders (such as low back pain, neck pain, and patellar tendinopathy) and explored the mechanical properties of soft tissue in these patients (Ishikawa et al., 2017; Breda et al., 2020; Koppenhaver et al., 2020). One study has investigated quadriceps tendon stiffness in patients with knee OA and they found the passive stiffness of the quadriceps tendon was negatively correlated to the maximum knee flexion angle in patients with knee OA and speculated that the increased soft tissues stiffness may contribute to functional impairment (Ebihara et al., 2020). Although patients with knee OA often experience pathological changes in the muscles around the knee (Rice et al., 2011; Noehren et al., 2018), to the best of our knowledge, no studies have investigated the muscles stiffness in patients with knee OA. Therefore, it is necessary to directly compare the differences in quadriceps stiffness between the healthy subjects and patients with knee OA to obtain a comprehensive understanding of the biomechanical properties of the muscle and to develop an appropriate rehabilitation program for patients with knee OA.

Quantitative assessment of muscle stiffness usually uses biomechanical methods to evaluate changes in the muscle-tendon length-tension relationship (Rieder et al., 2016). However, it evaluates the stiffness of the entire muscle group and cannot assess changes in the stiffness of individual muscles. A handheld device, MyotonPRO, can measure changes in individual muscle stiffness conveniently and quickly (Chang et al., 2020; Amirova et al., 2021). In our previous studies, we demonstrated that MyotonPRO is a reliable method for assessing the stiffness of the gastrocnemius (Feng et al., 2018) and upper trapezius (Liu CL et al., 2018). Chen et al. (2019) observed good intra- and interrater reliability of MyotonPRO for measuring the stiffness of the superficial quadriceps [vastus lateralis (VL), vastus medialis (VM) and rectus femoris (RF)] (ICC >0.84). Therefore, we compared the differences in the quadriceps stiffness between healthy people and patients with Knee OA using MyotonPRO.

The objectives of this study were to 1) compare the stiffness of the superficial quadriceps (RF, VL, and VM) between healthy individuals and patients with knee osteoarthritis; 2) examine differences of quadriceps stiffness at different angles of the knee joint; and 3) evaluate the correlations between the quadriceps (RF, VL, and VM) stiffness and joint dysfunction in patients with Knee OA.

## Materials and Methods

### Subjects

This study had a cross-sectional design. Twenty-five patients with knee OA and 25 healthy, asymptomatic, age-matched subjects were recruited for this study. The sample size was calculated based on a pilot study of 14 subjects. The effect size between the patients with knee OA and healthy controls for VL stiffness was 0.77. Taking *α* at 5% and power at 80%, the estimated sample size was 22 subjects per group. All patients applied to outpatient clinics with knee pain and received an initial clinical assessment (including knee X-rays) to support the clinical diagnosis of knee OA. The patients were included if they met the following criteria (Vaz et al., 2013; Devrimsel et al., 2019): 1) Age greater than 45 years old; 2) clinically diagnosed with knee OA; 3) patients diagnosed with grade 2 or 3 knee osteoarthritis according to the criteria proposed by Kellgren and Lawrence; 4) visual analog scale (VAS) > 3 points in daily activity; and 5) no skin lesions above the measuring regions. Patients’ exclusion criteria for this study were based on the following factors: a history of knee or hip or ankle surgery, previous musculoskeletal or joint injuries of lower limb in addition to knee OA, acute inflammation or pain with edema, metabolic diseases, severe deformity of the lower limbs, and BMI >30 kg/m^2^.

### Equipment

In the present study, MyotonPRO (Myoton AS, Tallinn, Estonia) was used to quantify the quadriceps stiffness. The device’s basic principles are as follows (Gavronski et al., 2007; Schneider et al., 2015): five short mechanical impulses (the tap interval was 0.8 s) were implemented automatically by the device after precompressing the tissue, and these impulses cause mechanical oscillations in the soft tissue being evaluated. Then, MyotonPRO recorded the oscillation information and calculated the soft tissue mechanical parameters. One of these parameters is stiffness (newtons/meter, N/m). The stiffness value was calculated as the maximum acceleration of the oscillation/maximum displacement of the tissue. The larger the value, the stiffer the tissue. Any data with a coefficient of variation greater than 3% in any measurement on quintuple scanning mode were remeasured.

### Procedures

Demographic information such as age, sex, weight, height, and BMI were recorded before the experiment. The Western Ontario and McMaster Universities Osteoarthritis Index (WOMAC) was used to assess the severity of the symptoms and physical functional disability among the knee OA patients (Salaffi et al., 2003). The questionnaire included 24 questions divided into three subscales: pain, stiffness and physical function. Each question was answered based on a validated 10-point numerical rating scale. The WOMAC has demonstrated acceptable validity and reliability in individuals with Knee OA (Bellamy et al., 1988). The total WOMAC scores were defined as the sum of 24 items, ranging from 0 to 240.

### Measurement of the Quadriceps Stiffness

The room temperature was maintained at 25°C throughout all tests. The quadriceps was subdivided into the rectus femoris (RF), vastus lateralis (VL), vastus medialis (VM), and vastus intermedius (VI). Because the VI is deep inside the RF, the stiffness of the VI cannot be measured by the MyotonPRO. According to previous studies, the measurement region for RF stiffness was two-thirds of the length between the anterior superior iliac spine (ASIS) and the superior pole of the patella (Agyapong-Badu et al., 2016; Chen et al., 2019). The stiffness of the VL and VM was measured at the most salient point of the muscle belly (near the knee joint) (Chen et al., 2019). The measurement sites were marked by the same experienced physical therapist. The symptomatic knees of the patients with knee OA were used for all measurements. When both knees were symptomatic, the most affected knee was evaluated (León-Ballesteros et al., 2020). We measured the stiffness of the soft tissues in the dominant legs in healthy participants. The dominant leg of the subject was determined by which leg they used when they were asked to kick a ball (Lenskjold et al., 2015).

Before the stiffness assessment, the participants were allowed to rest for 5 min. The stiffness measurement was taken with the participant in the sitting position with the knee bent at 60° and 90°. The knee angle was maintained by an angle-adjustable knee orthosis. The order of stiffness measurements was RF, VL, and VM. The MyotonPRO was applied perpendicular to the surface of the muscle being examined. The subjects were asked to refrain from talking, to remain relaxed, and to avoid any muscle contraction during the stiffness measurements.

### Statistical Analysis

SPSS Version 22.0 software (IBM, Armonk, NY, United States) was used for the data analysis. The demographic information was calculated by descriptive statistics. The Shapiro–Wilk test was used to assess the normal distribution of the data. Homogeneity of variances was tested using Levene’s test. Independent t tests were performed to compare the demographic data between individuals with and without knee OA. Comparisons between RF, VL, and VM stiffness in the healthy subjects and the patients with knee OA were evaluated using an independent sample *t*-test. A paired-sample *t*-test was performed for quadriceps stiffness differences at different knee angles. The correlation between RF, VL, VM stiffness, and WOMAC scores was demonstrated by Pearson correlation analysis (r). All measurement data are expressed as the mean ± standard deviation, and all *p* < 0.05 indicated a significant level.

## Results

### Demographic Information

Demographic information for all participants regarding age, weight, height, and BMI is depicted in Table 1. The clinical assessment report regarding WOMAC is also presented in Table 1. There were no significant differences in age, height, weight, or BMI (*p* > 0.05).

**TABLE 1:** The characteristics of the subjects.

Women/Men (n)	Patients with knee OA (M ± SD)	Healthy subjects (M ± SD)	*p*
	17/8	17/8	
Age (years)	62.20 ± 8.30	59.44 ± 5.33	0.168
Height (m)	1.62 ± 0.06	1.63 ± 0.06	0.873
Weight (kg)	63.92 ± 7.14	62.64 ± 8.13	0.557
BMI (kg/m^2^)	24.22 ± 1.96	23.67 ± 2.67	0.55
WOMAC	103.48 ± 27.73	—	—

WOMAC, the Western Ontario and McMaster Universities Osteoarthritis Index scores.

### RF, VL, and VM Stiffness Between the Patients With Knee OA and Healthy Subjects

The mean stiffness values of the RF, VL and VM in the patients with knee OA and healthy controls are summarized in Table 2. The VL stiffness of patients with knee OA was greater than that of the healthy subjects at flexion 60° of the knee joint (*p* < 0.05). Similarly, compared with the healthy subject group, the patients in the knee OA group had greater VL stiffness at 90° of knee flexion (*p* < 0.05). However, no between-group differences were observed in the RF and VM stiffness measured at 60° and 90° of knee flexion (*p* > 0.05).

**TABLE 2:** Stiffness of the RF, VL, and VM between the patients with Knee OA and the healthy subjects.

Knee flexion		Patients with knee OA (M ± SD)	Healthy subjects (M ± SD)	*p*
60°	RF	268.68 ± 37.21	262.96 ± 31.10	0.558
	VL	288.80 ± 29.78	254.88 ± 29.33	0.001^**^
	VM	260.92 ± 30.68	246.80 ± 30.56	0.110
90°	RF	292.48 ± 37.86	286.32 ± 34.42	0.987
	VL	321.92 ± 27.47	289.88 ± 26.81	0.001^**^
	VM	290.36 ± 39.22	291.40 ± 40.07	0.926

RF, rectus femoris; VL, vastus lateralis; VM, vastus medialis. **p < 0.05.

### RF, VL, and VM Stiffness at Different Degrees of Knee Flexion

Figures 1, 2 reveal the stiffness of RF, VL, and VM at 60° and 90° of knee flexion in patients with knee OA and healthy subjects, respectively. A significant difference was found in the RF, VL, and VM stiffness between the 60° of knee flexion and 90° flexion of the knee joint in the patients with knee OA (*p* < 0.05). Similarly, in the healthy subject group, there was a significant increase in the RF, VL, and VM stiffness at 90° flexion of the knee joint compared with that at 60° of knee flexion (*p* < 0.05).

**FIGURE 1:** The difference between the mean stiffness of the quadriceps at 60° and 90° of knee flexion in patients with knee OA. **p < 0.05.

**FIGURE 2:** The difference between the mean stiffness of the quadriceps at 60° and 90° of knee flexion in healthy subjects. **p < 0.05.

### The Correlation Between RF, VL, VM Stiffness, and WOMAC Scores

In patients with Knee OA, Pearson correlation analysis tests were used to indicate the relationship between RF, VL, VM stiffness, and WOMAC scores. As shown in Table 3, there was a significant positive correlation (*r* = 0.508, *p* = 0.010) between the WOMAC scores and the VL stiffness measured at 60° of knee flexion. At 90° of knee joint flexion, a significant positive correlation was found between the WOMAC scores and the VL stiffness (*r* = 0.456, *p* = 0.022). However, no significant correlation was apparent between RF and VM stiffness and WOMAC scores, regardless of knee position (*p* > 0.05). The stiffer the VL is, the greater the level of physical dysfunction in knee OA patients.

**TABLE 3:** Correlation of RF, VL, and VM stiffness and WOMAC scores.

Knee flexion		WOMAC	
		r	*p*
60°	RF	0.297	0.149
	VL	0.508	0.010^**^
	VM	0.284	0.169
90°	RF	0.283	0.170
	VL	0.456	0.022^**^
	VM	0.328	0.110

RF, rectus femoris; VL, vastus lateralis; VM, vastus medialis; WOMAC, the Western Ontario and McMaster Universities Osteoarthritis Index scores. **p < 0.05.

## Discussion

This is the first study to compare the stiffness of the VL, RF and VM between subjects with Knee OA and healthy controls. The present study aimed to investigate the difference in the stiffness of the VL, RF and VM between subjects with and without knee OA. The main results of the study demonstrated that increased VL stiffness was found in subjects with knee OA compared to healthy controls. Furthermore, the findings from this study revealed that the quadriceps stiffness increased with knee flexion. More importantly, our study also established a relationship between the stiffness of the VL, RF and VM and the degree of disability among subjects with knee OA. We found a significant positive correlation between the VL stiffness index and WOMAC scores.

We observed the VL stiffness among subjects with Knee OA was higher than that among healthy controls. The VL stiffness was increased by 11.8% at 60° of knee flexion and by 10.0% at 90° of knee flexion compared to the control group. Although no previous studies have made a direct comparison as in our study, previous studies have reported that a reduction in muscle flexibility may be associated with anterior knee pain (Witvrouw et al., 2000; Piva et al., 2005). A 2-year prospective study revealed that there was significantly less flexibility of the quadriceps in subjects with patellofemoral pain (Witvrouw et al., 2000). They found that the flexibility of the quadriceps in subjects with patellofemoral pain was reduced by 6.1% compared to the control group. Similarly, Piva et al. (2005) observed that patients with patellofemoral pain syndrome had a reduced knee range of motion. In the study of Witvrouw et al. (2001), significantly lower flexibility of the quadriceps in individuals with patellar tendinitis was obtained as compared with the control group (Witvrouw et al., 2001). A recent study evaluated the stiffness of the RF and VL in athletes with patellar tendinopathy using shear wave elastography, and they observed that the VL stiffness was increased by 26.5% in athletes with patellar tendinopathy (Zhang et al., 2017). More recently, Zhou et al. (2020) reported that a stiffer medial gastrocnemius but not the lateral gastrocnemius was found in individuals with plantar fasciitis. The knee extensor plays an important role in dissipating kinetic energy during walking, running and landing (Decker et al., 2003), and a decrease in the flexibility of the quadriceps muscle might contribute to increasing the loading on the patellofemoral joint (Piva et al., 2005). Some studies have investigated the effects of soft tissue release in patients with knee OA (Tarabichi and Tarabichi, 2010; Atkins and Eichler, 2013). Atkins and Eichler, 2013 conducted a randomized controlled trial and observed a significant difference in the WOMAC score between the self-massage intervention group (applied on the quadriceps) and the control group after intervention. And Field (2016) suggested the massage therapy on quadriceps and hamstrings could reduce pain and increase the knee ROM. Tarabichi and Tarabichi (2010) also found a significant increase in knee ROM after quadriceps release alone in patients with knee OA. The findings from the present study indicate that releasing the quadriceps (especially VL muscle) may have a positive effect on the prevention and treatment of patients with knee OA. Therefore, additional studies need to be conducted to investigate the effectiveness of releasing the tightness of the VL for subjects with knee OA.

As shown in Figure 1 and Figure 2, the stiffness of RF, VL, and VM in 90° flexion of the knee joint was significantly higher than that in 60° flexion of the knee, regardless of whether patients with knee OA or healthy subjects were included. Similarly, Coombes et al. (2018) reported that the stiffness of the quadriceps muscle quantified with shear wave elastography increased with knee flexion. Xu et al. (2018) observed that the passive tension of RF, VL and VM started to increase at 51°, 48°, and 45° flexion, respectively, of the knee joint in rowers (Xu et al., 2018). These cases demonstrate the straining-stiffening behavior of soft tissue after the fibers become tight (DeWall et al., 2014). Chen et al. (2019) measured the stiffness of RF, VL and VM in young healthy participants at different angles of knee flexion using MyotonPRO, and they observed an increase of 11.38 and 18.59% in VL stiffness and VM stiffness in the nondominant limb from 60° to 90° flexion of the knee, respectively, while there was no significant difference in RF stiffness. Their results for VL and VM stiffness are similar to our results. In the present study, changing from 60 to 90° flexion of the knee resulted in 13.73 and 18.07% VL and VM stiffness in the control group, respectively, but we also found an increase of 8.88% in RF stiffness. Possible reasons for different variations in RF stiffness measurements may include the different measurement methodologies and the differences in the participants being studied.

In the present study, we also detected a positive correlation between VL stiffness and WOMAC scores in patients with knee OA. To the best of our knowledge, this is the first study to investigate the correlation between quadriceps stiffness and the level of function of patients with knee OA. Some previous studies also focused on the correlations between soft tissue stiffness and pain intensity or the functional level of the patients (Zhang et al., 2014; Koppenhaver et al., 2020; Zhou et al., 2020). In the study of Koppenhaver et al. (2020), lumbar muscle stiffness was greater in individuals with low back pain than in asymptomatic participants and was associated with pain intensity as quantified with the numeric pain rating scale and the level of disability measured by the Oswestry Disability Index (Koppenhaver et al., 2020). Zhou et al. (2020) observed that the stiffness of the medial gastrocnemius was positively correlated with pain intensity in patients with plantar fasciitis. Significant correlations were found between the elastic properties of the patellar tendon and pain and dysfunctions in athletes with patellar tendinopathy (Zhang et al., 2014). The above evidence indicates that soft tissue stiffness may be related to some functional outcomes in patients with musculoskeletal disorders. Chino and Takahashi et al. (2015) and Chino and Takahashi et al. (2016) found that increased muscle stiffness can contribute to an increase in passive joint stiffness. Miyamoto and Hirata (2019) found that muscle stiffness was negatively correlated with joint ROM. Ebihara et al. (2020) investigated the correlation between the passive stiffness of the quadriceps tendon and the gait parameters in the swing phase during gait, and they found that there was a negative correlation between the stiffness of the quadriceps tendon and gait speed and step length in patients with knee OA. Therefore, we speculate that the positive correlation between VL stiffness and WOMAC scores may be caused by the increased VL stiffness leading to decreased knee ROM or increased knee joint stiffness or further increased difficulty in performing activities of daily living in patients with knee OA.

There are some limitations of this study. First, only one point each in the RF, VL and VM was assessed, and our findings could not be generalized to other regions of the quadriceps muscle. Second, although we suggested that subjects be completely relaxed during the stiffness measurements, electromyography was not used to monitor the quadriceps muscle activity and ensure it was not firing. Third, the order of stiffness measurement of quadriceps was not randomized, which may introduce potential bias. In addition, due to the limitations of MyotonPRO, we did not investigate the stiffness of the vastus intermedius. Finally, this study indicated that the VL stiffness was related to the WOMAC score. However, it was not clear whether the VL stiffness affected the level of function in patients with knee OA. A prospective study is necessary to ascertain the cause and effect relationship between passive muscle stiffness and the degree of function in patients with knee OA.

## Conclusion

Patients with knee OA have an increase in the stiffness of the vastus lateralis, and the stiffness of the quadriceps is increased with knee flexion in individuals with and without knee OA. In addition, the stiffness of the vastus lateralis is associated with the WOMAC score in patients with knee OA.

## Data Availability

The raw data supporting the conclusion of this article will be made available by the authors, without undue reservation.
